The article "Lactobacillus paracasei X11 Ameliorates Hyperuricemia and Modulates Gut Microbiota in Mice" was retracted in 2024. Reason: duplicated data.

# *Lactobacillus paracasei* X11 Ameliorates Hyperuricemia and Modulates Gut Microbiota in Mice

**DOI:** 10.3389/fimmu.2022.940228

**Published:** 2022-07-06

**Authors:** Jiayuan Cao, Qiqi Liu, Haining Hao, Yushan Bu, Xiaoying Tian, Ting Wang, Huaxi Yi

**Affiliations:** College of Food Science and Engineering, Ocean University of China, Qingdao, China,

**Keywords:** hyperuricemia, uric acid-lowering, *Lactobacillus paracasei* X11, gut microbiota, ameliorating

## Abstract

Hyperuricemia (HUA) is the presence of excessive uric acid (UA) in blood, which leads to an increased risk of chronic kidney disease and gout. Probiotics have the potential effect of alleviating HUA. The purpose of this study was to screen probiotics with UA-lowering activity and explore the underlying mechanism. The UA-lowering activity of 20 lactic acid bacteria strains was investigated *in vitro*, and the effect of candidate probiotics on UA metabolism was evaluated using the HUA Balb/c mouse model. The results showed that *Lactobacillus paracasei* X11 had excellent UA-lowering activity *in vitro*, which could degrade nucleotides and nucleosides completely within 30 min, and the degradation rates of purine and trioxypurine could reach 83.25% and 80.42%, respectively. In addition, oral administration of *L. paracasei* X11 could reduce serum UA by 52.45% and inhibit renal proinflammatory cytokine IL-1β by 50.69%, regulating adenosine deaminase (ADA), xanthine oxidase (XOD), and transporter expression (GLUT9, NPT1, and URAT1) to a normal level. Moreover, it could restore the ratio of *Bacteroidetes* to *Firmicutes* (Bac/Firm ratio) and showed a positive effect on the recovery of the intestinal microbiota. These findings provided fundamental information about the UA-lowering properties of probiotics, which suggested that *L. paracasei* X11 had the potential to be developed as a novel probiotic strain to ameliorate HUA.

## Introduction

Hyperuricemia (HUA) is an idiopathic inflammatory disease characterized by a long-term purine metabolism disorder and persistently elevated blood uric acid (UA) concentration (1–3). In clinical practice and research, HUA is generally reported when the serum urate is above 0.42 mmol/L (7 mg/dl) for men or 0.36 mmol/L (6 mg/dl) for women (4). It may result in the deposition of UA crystals, which promotes high comorbidity burden and finally leads to tissue damage such as gout (5), atherosclerosis (6), type 2 diabetes mellitus (7), vascular damage (8), and chronic kidney disease (9). The incidence of HUA has been remarkably increased by about 20% worldwide (10), and the patients have become younger, which is of concern (11, 12), so HUA has emerged as a public health challenge.

UA is an antioxidant product of purine metabolism in the body, which is beneficial to humans in proper amounts (1). Urate homeostasis depends on the balance between its production in the liver and the excretion in the kidney and intestine (8). Because of the lack of uricase in the human body that converts urate into water-soluble allantoin (13, 14), the generated UA cannot be further readily eliminated. When the balance between production and excretion of UA is lost, it may bring about the excessive internal deposition of urate crystal (15, 16). Environmental exposures including purine-rich foods (5) (such as seafood, beer, and red meat) and sub-healthy physical states under excessive pressure also give rise to high levels of UA in plasma. The existing treatment methods for HUA include drug therapy and non-drug therapy, but all of them have adverse effects such as changing dietary habits, nutritional imbalance, side effects such as kidney stones, and all-cause cardiac death (17). Based on the defects and deficiencies of existing treatment, it is urgent to seek a strategy with obvious effect, stability, safety, and convenience for HUA.

Probiotics have been confirmed as active microorganisms, which can provide positive health effects to the host (18). Microbial remediation has been widely accepted by the public as a cost-effective treatment because of minimum lesions in humans (19, 20). At the same time, intestinal microbiota has been reported to exert significant impacts on metabolic diseases (20–22), including modulation of the immune system (21, 22) and protection against pathogens (23). Guo et al. found that *Bacteroides caccae* and *Bacteroides xylanisolvens* were rich in the intestinal tract of HUA patients, while *Faecalibacterium prausnitzii* and *Bifidobacterium pseudocatenulatum* were absent significantly (17, 19, 24). Probiotics can mitigate this imbalance of intestinal microbiota and compensate for the side effects of drugs (17, 19).

In this study, the probiotics with uric-lowering activity were screened *in vitro* firstly, then the uric-lowering activity was verified by the HUA mouse model *in vivo*, and the underlying mechanism was explored from the viewpoint of gut microbiota. This study will lay the foundation for the development of probiotics to prevent or ameliorate HUA and provide a novel treatment strategy for HUA patients.

## Materials and Methods

### Strain Cultivation

Twenty lactic acid bacteria strains were isolated from traditional fermented food such as yak yogurt and pickles and stored in glycerin at −80°C. In MRS liquid medium (QingDao Hopebio Technology, Qingdao, China), 2% (v/v) strains were inoculated and cultured at 37°C for 24 h. Optical density (OD) was measured at 600 nm to determine the growth state for use.

### Determination of Nucleoside Degradation Activity *In Vitro*

After the subculture was generated 3 times, the fermentation broth was centrifuged at 5,000 rpm at 4°C for 10 min to obtain sediments, which were washed with 1 ml of phosphate-buffered saline (PBS) 3 times, and then suspended in 1 ml of uric-neutral potassium phosphate solution, purine-neutral potassium phosphate solution, nucleoside-neutral potassium phosphate solution, and nucleotide-neutral potassium phosphate solution (100 mmol/L, pH = 7). The mixed solution was cultured under anaerobic conditions at 37°C for 30 min. Then the terminator perchloric acid was added at 9:1 (v/v), and the mixture was filtered through 0.22-μm filters. Filtered solution measuring 20 μl was taken for high-performance liquid chromatography (HPLC) analysis (chromatographic column, ZORBAX Eclipse Plus C18, 4.6 × 250 mm, 5 μm; column temperature, 25°C; UV detection wavelength, 254 nm; mobile phase, 20 mmol/L of isogradient phosphate buffer solution; flow rate, 1 ml/min; elution time, 45 min). The degradation rate of nucleosides was calculated according to the following formula.


$$Degradation\;Rate\;\left(\%\right)=\frac{\left(C_{Standard}-C_{Sample}\right)}{C_{Standard}}*100\%$$

### Animals and Experimental Design

Specific pathogen-free (SPF) Balb/c mice (male; 6 weeks of age) were purchased from Beijing Weitong Lihua Experimental Animal Technology Co., Ltd. (Animal Qualification Certificate Number: SCXK (Beijing) 2014-0001). Mice were housed at 18°C–24°C in 12-h light/dark cycles, and the relative humidity of the animal room was 50%–70%. The mice were acclimatized for 1 week before use. All animals were maintained in individual cages, and the total experimental duration was 5 weeks. The experiment was conducted in accordance with the animal management regulations of the Ministry of Science and Technology of China and approved by the Experimental Animal Ethics Committee of the College of Food Science and Engineering, Ocean University of China (Permission number: SPXY2022011201).

The mice were randomly assigned to 4 groups: control group (CON), model group (MOD), probiotics group (X11), and active drug control group (ADC). The establishment of the HUA model is shown in **Figure 1**. The CON group was fed a normal diet and water, and the other groups were fed a high-purine diet (containing 400 g/kg of yeast extract, 20 g/kg of ribonucleic acid, and fructose water). To induce HUA, the mice were intraperitoneally injected with 400 mg/kg of potassium oxazinate dissolved in 0.5% CMC-Na solution for 4 weeks. After successful modeling, intragastric administration of 10 ml/kg body weight was started. The CON and MOD group were given 0.85% NaCl, the X11 group was given 10^9^ CFU/ml of *Lactobacillus paracasei* X11, and the ADC group was given 42 mg/kg of allopurinol (ALLO). Blood samples were collected from the eyeball veins of mice on the 7th, 21st, and 35th days. Hepatic, renal, and intestinal tissues were collected and stored at −80°C until use.

**Figure 1:** Experimental chart of *Lactobacillus paracasei* X11 in treatment of HUA mice. HUA, hyperuricemia.

### Body Weight and Organ Coefficient Measurement

The body weight of mice was monitored and recorded. The weight of the whole kidney and liver were also recorded, and the organ index was calculated according to the following formula (25).


$$Liver\;Index\;\left(\%\right)=\frac{M_{Liver}}{M_{Body}}*100\%$$

$$Kidney\;Index\;\left(\%\right)=\frac{M_{Kidney}}{M_{Body}}*100\%$$

### Serum Analyses

Blood samples were placed for 2 h and centrifuged to obtain the supernatant. The serum levels of UA, blood urea nitrogen (BUN), creatinine (Cr), and xanthine oxidase (XOD) were measured by ELISA kits (Suzhou Kaerwen, Suzhou, China).

### Histopathological Examination

The histopathological examination was performed according to the report of Wu et al. (19) with minor modifications. In 4% paraformaldehyde, 1-cm mouse ileum tissue and 0.8 × 0.8 cm mouse liver and kidney tissue samples were fixed for 24 h and then embedded in paraffin. A piece was cut from the paraffin block (4 μm thick) and H&E-stained. The stained sections were observed under an optical microscope (E100, Nikon) and photographed.

### Inflammation Cytokine Detection

Liver and kidney tissue samples were homogenized in 0.9% cold saline and then centrifuged at 5,000 rpm for 10 min to obtain the supernatant. The levels of interleukin-1β (IL-1β), tumor necrosis factor-α (TNF-α), and malondialdehyde (MDA) in homogenate and the concentration of IL-1β and lipopolysaccharide (LPS) levels in the serum were determined using commercial ELISA kits (Suzhou Kaerwen, China) according to the manufacturer’s instructions.

### Hepatic Metabolism Enzyme Determination

The hepatic tissue was homogenized by a high-speed lapping instrument (Shanghai, China) and stored in a refrigerator at −80°C until use. The hepatic metabolism enzyme adenosine deaminase (ADA) and XOD were detected by the ELISA kit (Suzhou Kaerwen, China) according to the manufacturer’s instructions.

### Real-Time PCR Assay

The mRNA expression levels of glucose transporter 9 (GLUT9), sodium-phosphate cotransporter type 1 (NPT1), and urate transporter 1 (URAT1) were evaluated *via* RT-PCR. Tissue samples measuring a total of 50 mg were homogenized in 1 ml of TRIzol lysate (Biosharp, Hefei, China) to extract the total RNA. Then, cDNA was synthesized using the 5× All-In-One RT MasterMix reverse transcription reaction kit (ABM, Richmond, BC, Canada). Forward and reverse primer sequences were synthesized by Sangon Biotech Co. Ltd. (Shanghai, China) in **Table 1**. The 2^−ΔΔCt^ method was utilized to normalize the expression results.

**Table 1:** Target gene primer sequences.

Gene	Forward (5′–3′)	Reverse (5′–3′)
β-Actin	ACTGCTCTGGCTCCTAGCAC	CCACCGATCCACACAGAGTA
GLUT9	ATGTGGACTCAATGCGATCTGGTTC	TGTTTCAATTCCTCCCGTGCTCAG
NPT1	TGTTGGGTGTGTTCTGAGTCTTTCC	CCTTCTCACTGCTGCTCATATACGG
URAT1	GACCTTGGACCCGATGTTCTTCTG	CGTGGCGTTGGACTCTGTAAGC

### 16S rRNA Gene Sequencing

The fecal samples were collected from individually housed mice on the last day of intragastric treatment and then underwent immediate freezing at −80°C. When the genomic DNA was extracted by Fast DNA SPIN extraction kits (Santa Ana, CA, USA), it was further used as the template to amplify the 16S rRNA gene by Q5 High Fidelity DNA Polymerase. The variable V3–V4 regions of the 16S rRNA gene were amplified using the forward primer 338F (ACTCCTACGGGAGGCAGCA) and the reverse primer 806R (TCGGACTACHVGGGTWTCTAAT). PCR amplicon was purified and quantified and then sequenced by Shanghai Personal Biotechnology Co., Ltd. (Shanghai, China).

### Statistical Analysis

All data were expressed as the mean ± SD, and all analyses were performed in triplicate. One-way ANOVA and Duncan’s test for multiple comparisons were performed by SPSS (Version 22.0) to analyze the differences among the groups, which are shown with asterisks or letters.

## Results

### Screening of Lactic Acid Bacteria With Uric Acid-Lowering Activity

The assimilating ability of nucleotide, nucleoside, purine, and trioxypurine of 20 lactic acid bacteria strains isolated from Chinese traditional fermented food was assayed by HPLC. The results are summarized in **Table 2**. It was shown that *L. paracasei* X11 exhibited an excellent assimilation rate, which could completely degrade nucleotides and nucleosides within 30 min, and the degradation rates of purine and trioxypurine could reach 83.25% and 80.42%, respectively (*p* < 0.05). In addition, in our previous study, *L. paracasei* X11 was found to have good gastrointestinal viability, such as surface hydrophobicity and self-aggregation, acid and bile salt resistance, and gastric and intestinal juice tolerance (26).

**Table 2:** Quantitative determination of UA-lowering activity of the strains.

Strain	Nucleotide degradation rate (%)	Nucleoside degradation rate (%)	Purine degradation rate (%)	Uric acid degradation rate (%)
FN2-39	68.1484 ± 1.9597	76.0759 ± 2.5828	72.6720 ± 1.1685	40.7223 ± 2.5316
J5	92.9175 ± 1.9205	81.1367 ± 4.7229	57.7971 ± 5.0708	44.4617 ± 0.7307
M3-2-1	64.5186 ± 5.0598	79.4009 ± 1.1137	66.2683 ± 0.5522	21.0915 ± 9.9491
FN518	80.2143 ± 1.6908	79.2538 ± 1.1992	67.8075 ± 2.8154	57.0609 ± 2.3926
KV9	87.3277 ± 4.7697	85.7095 ± 4.4631	69.3296 ± 6.8912	28.0097 ± 1.9478
MDHXM	92.5765 ± 0.1819	89.4102 ± 1.9665	66.8331 ± 2.1358	6.9196 ± 4.0219
X11	99.9965 ± 0.0011	99.9987 ± 0.0023	83.2462 ± 0.9644	80.4153 ± 1.8229
K11	70.1502 ± 5.0934	88.5926 ± 4.9378	76.6868 ± 0.4113	42.2661 ± 3.1298
YR3115	37.2716 ± 2.1795	81.5065 ± 3.1096	73.3516 ± 2.2941	38.8039 ± 2.9163
F1-7	76.6291 ± 8.3031	82.7201 ± 4.5419	60.6868 ± 2.4632	29.2897 ± 3.0150
MN45	58.2545 ± 0.1023	64.7772 ± 3.1109	64.8054 ± 0.6875	50.5192 ± 2.9395
F27-3	69.2139 ± 8.1247	68.1975 ± 6.9705	36.5312 ± 1.3944	49.1143 ± 3.7025
MN20	48.4488 ± 2.3413	45.1674 ± 1.5165	58.0608 ± 4.3048	57.3631 ± 2.6593
YZX-21	73.3027 ± 2.2671	65.6776 ± 1.8260	52.7699 ± 2.8804	41.8382 ± 1.5089
1F-6	71.7534 ± 2.4152	79.8313 ± 1.3130	18.8075 ± 6.2836	26.3679 ± 2.2030
MFGSQ	76.2463 ± 0.0179	80.2348 ± 1.5708	38.3278 ± 8.9261	-6.5966 ± 5.1704
L-577	70.6311 ± 8.4608	78.9717 ± 2.0439	68.8700 ± 2.2448	34.8002 ± 4.8300
LGG	73.2782 ± 0.7263	79.8248 ± 1.0010	58.1199 ± 4.8671	26.9346 ± 1.3504
YZX-38	78.3186 ± 8.5527	78.8045 ± 1.1141	67.4593 ± 2.1933	32.7707 ± 3.8295
F1-3-2	72.8688 ± 0.5476	77.4971 ± 8.4655	12.1073 ± 1.0656	15.9451 ± 2.5814
FN2-39	68.1484 ± 1.9597	76.0759 ± 2.5828	72.6720 ± 1.1685	40.7223 ± 2.5316
J5	92.9175 ± 1.9205	81.1367 ± 4.7229	57.7971 ± 5.0708	44.4617 ± 0.7307
M3-2-1	64.5186 ± 5.0598	79.4009 ± 1.1137	66.2683 ± 0.5522	21.0915 ± 9.9491

UA, uric acid.

### Determination of Body Weight and Organ Index of Mice

According to the experimental results of UA-lowering activity *in vitro*, *L. paracasei* X11 was selected to explore the UA-lowering activity *in vivo*. As shown in **Table 3**, there was no statistical difference in the weight of mice at baseline. However, the weight gain of the mice in the CON group and X11 group was significantly higher than that of the MOD group and ADC group after 4 weeks (*p* < 0.05). It was found that the liver weight, liver index, kidney weight, and kidney index of the MOD group were significantly higher than those of the CON group (*p* < 0.05). The liver index of the MOD group increased by 28.85% as compared with the CON group (*p* < 0.05). Compared with those of the MOD group, the liver and kidney index of the X11 group decreased by 0.35% and 6.32%, respectively (*p* < 0.05). The renal coefficient of the ADC group was significantly higher than that of the MOD group by 6.9% (*p* < 0.05).

**Table 3:** Effects of *Lactobacillus paracasei* X11 on body weight, organ coefficient in hyperuricemia mice.

Group	Initial weight/g	Final weight/g	Liver weight/g	Liver index/%	Kidney weight/g	Kidney index/%
CON	20.70 ± 0.82^a^	24.21 ± 1.08^b^	1.04 ± 0.02^a^	4.29 ± 0.22^a^	0.35 ± 0.02^a^	1.47 ± 0.11^a^
MOD	20.54 ± 0.63^a^	23.13 ± 1.13^a^	1.34 ± 0.08^bc^	5.74 ± 0.40^a^	0.41 ± 0.07^b^	1.74 ± 0.27^bc^
X11	20.66 ± 0.91^a^	24.33 ± 1.00^b^	1.39 ± 0.11^c^	5.72 ± 0.40^a^	0.40 ± 0.04^ab^	1.63 ± 0.15^ab^
ADC	20.79 ± 0.93^a^	21.85 ± 1.15^c^	1.21 ± 0.20^b^	5.56 ± 1.00^b^	0.41 ± 0.03^b^	1.86 ± 0.10^c^

CON, control; MOD, model; X11, probiotics; ADC, active drug control.

Identical letters represent no significant difference and different letters represent significant difference. (P < 0.05).

### Effect of *Lactobacillus paracasei* X11 on Histopathological Changes

As shown in **Figure 2**, it was observed that the morphology of hepatocytes in the CON group was normal while it was swollen in the MOD group. The cytoplasm turbidness was severe, and the fatty vacuole depositions were obvious in the MOD group, which were alleviated in the X11 group and ADC group. However, the glomerulus in the MOD group and ADC group was atrophic and deformed, and the renal tubule lumen was dilated significantly compared with the CON group. *L. paracasei* X11 could improve the above adverse symptoms and reduce inflammatory cell infiltration. The villi in the MOD group and ADC group became shorter and were distributed sparsely. Conversely, the villi length and the crypt depth ratio in the X11 group were improved, and the lipid infiltration and the damage caused by UA and ALLO were alleviated.

**Figure 2:** Histopathological analyses of H&E-stained liver and kidney sections (×200 magnification) and intense sections (×100 magnification) from mice.

### Examination of Serum Biochemical Indicators

To examine the effect of the *L. paracasei* X11 on the serum biochemical indicators of HUA mice, intraperitoneal injection of potassium oxonate and a supplement with a high purine diet were given to mice for 4 weeks. In **Figure 3**, it was found that the levels of UA, BUN, Cr, and XOD in serum of the MOD group were increased to 241.37 ± 14.51 μmol/L, 13.41 ± 0.54 mmol/L, 98.73 ± 12.48 μmol/L, and 2.71 ± 0.24 U/L, respectively. The concentration of these serum biochemical indicators was more than double that of the CON group (*p* < 0.05).

**Figure 3:** Effects of *Lactobacillus paracasei* X11 on serum biochemical indicators of mice. **(A)** UA. **(B)** BUN. **(C)** CRE. **(D)** XOD. UA, uric acid; BUN, blood urea nitrogen; CRE, creatinine; XOD, xanthine oxidase. The same number of asterisks indicates no significant difference and the different number of asterisks indicates significant difference. (P < 0.05).

After 14 days’ gavage, it was observed that the administration of *L. paracasei* X11 could reduce the levels of UA, BUN, Cr, and XOD in serum by 52.45%, 26.75%, 47.54%, and 44.60% compared with those of the MOD group, respectively (*p* < 0.05). The results showed that the levels of UA, BUN, and XOD in the ADC group were decreased, which were almost equal to those of the CON group and significantly lower than those of the MOD group (*p* < 0.05). However, the Cr level was increased by 115.74 ± 2.59 μmol/L in the ADC group compared with other groups (*p* < 0.05). These findings indicated that *L. paracasei* X11 possessed a potential therapeutic effect by reducing the serum biochemical indicators in HUA and avoiding the side effect of the clinical drug ALLO.

### Effects of *Lactobacillus paracasei* X11 on Proinflammatory Factors

To further analyze the effect of the *L. paracasei* X11 on the proinflammatory factors of mice, the levels of IL-1β, TNF-α, MDA, and LPS were assayed in **Figure 4**. An increasing trend of proinflammatory factors was observed in the MOD group (*p* < 0.05). Compared with the MOD group, the levels of serum IL-1β and LPS in the X11 group were decreased by 44.42% and 41.19%, respectively (*p* < 0.05). In the hepatic and renal homogenates, the concentration of IL-1β, TNF-α, and MDA in the MOD group was significantly increased but dropped after the intervention of *L. paracasei* X11 (*p* < 0.05). In the liver and kidney, the content of IL-1β reduced by 35.74% and 50.69%, the TNF-α content reduced by 48.31% and 48.29%, and the MDA content reduced by 31.96% and 33.36%, respectively (*p* < 0.05). Conversely, parts of these markers (IL-1β, TNF-α, MDA, and LPS) in the ADC group were further increased, which suggested that the side effect of ALLO exacerbated the inflammation in mice.

**Figure 4:** Effects of *Lactobacillus paracasei* X11 on proinflammatory factors of mice. **(A)** Serum IL-1β. **(B)** Serum LPS. **(C)** Liver IL-1β. **(D)** Kidney IL-1β. **(E)** Liver TNF-α. **(F)** Kidney TNF-α. **(G)** Liver MDA. **(H)** Kidney MDA. LPS, lipopolysaccharide; MDA, malondialdehyde. The same number of asterisks indicates no significant difference and the different number of asterisks indicates significant difference. (P < 0.05).

### Effects of *Lactobacillus paracasei* X11 on Uric Acid Metabolism Enzyme Activity

To evaluate the effect of the *L. paracasei* X11 on the activity of UA metabolism enzyme in mice, the levels of hepatic ADA and XOD were assayed and shown in **Figure 5**. It was observed that both ADA and XOD enzymatic activities in the MOD group were significantly increased compared with those of the CON group (*p* < 0.05). Alternatively, the enzyme vigor of ADA and XOD in the X11 group was inhibited, which was consistent with the ADC group. The enzyme activities of ADA and XOD were downregulated by 30.59% and 33.69%, respectively (*p* < 0.05), which indicated that *L. paracasei* X11 might reduce UA levels by inhibiting the activity of hepatic UA synthase.

**Figure 5:** Effects of *Lactobacillus paracasei* X11 on metabolism enzyme of mice. **(A)** Liver ADA. **(B)** Liver XOD. ADA, adenosine deaminase; XOD, xanthine oxidase. The same number of asterisks indicates no significant difference and the different number of asterisks indicates significant difference. (P < 0.05).

### Expression Level of Renal Re-Absorption and Excretion Transporter

To investigate the effect of *L. paracasei* X11 on the expression level of the transporter in mice, the renal re-absorption transporters GLUT9 and URAT1 and the excretion transporter NPT1 involved in UA metabolism were detected. As illustrated in **Figure 6**, compared with the CON group, the MOD group had no significant changes in the expressions of URAT1 and NPT1. Nevertheless, the GLUT9 level significantly increased in the MOD group (*p* < 0.05). Compared with the MOD group, the expressions of re-absorption transporters GLUT9 and URAT1 in the X11 group were decreased by 24.39% and 24.69%, respectively (*p* < 0.05), whereas the expression of excretion transporter increased by 7.3% (*p* < 0.05). In addition, *L. paracasei* X11 could maintain the relative mRNA to normal expression level, which was similar to that of the CON group.

**Figure 6:** Effects of *Lactobacillus paracasei* X11 on transporter expression level of mice. The same number of asterisks indicates no significant difference and the different number of asterisks indicates significant difference. (P < 0.05).

### Effects of *Lactobacillus paracasei* X11 on Gut Microbe in Hyperuricemia Mice

To explore the effect of *L. paracasei* X11 on the gut microbe of mice, the microbiota analysis of mouse fecal was performed by MiSeq sequencing of 16S rRNA. It was found that the diversity of gut microbial was decreased in the MOD group, which was moderately restored upon *L. paracasei* X11 treatment (**Figure 7A**). Specifically, a lower number of OTU was observed in the ADC group compared with that of the CON group and X11 group (**Figure 7B**). In addition, the α-diversity of the microbial community in different groups was comparatively studied. It was shown that the Goods_ coverage index was significantly decreased in the MOD group, whereas treatment with *L. paracasei* X11 restored the α-diversity of gut microbiota effectively (**Figure 7C**). The principal coordinates analysis (PCoA) suggested that *L. paracasei* X11 could shape the gut microbiota in HUA model mice and regulate it to a normal microbial community (**Figure 7D**).

**Figure 7:** Effects of *Lactobacillus paracasei* X11 on gut microbe of mice. **(A)** Results of the taxonomic annotation. **(B)** Venn diagram of ASV/OTU in the feces. **(C)** α-Diversity indexes calculated with QIIME2 according to ASV/OTU numbers of each group (*p* < 0.05). **(D)** β-Diversity evaluated using the weighted UniFrac-based PCoA. **(E)** Bar graphs showing the relative abundance of different bacteria at the phylum level. **(F)** Relative abundances of Bacteroidetes at the phylum level (*p* < 0.05). **(G)** Relative abundances of Firmicutes at the phylum level (*p* < 0.05). **(H)** Changes in the Bac/Firm ratio in the different groups (*p* < 0.05). **(I)** Bar graphs showing the relative abundance of different bacteria at the genus level. **(J)** Relative abundances of *Lactobacillus* at the genus level (*p* < 0.05). **(K)** Cladogram based on LEfSe analysis showing community composition of the gut microbiota in mice. **(L)** Linear discriminant analysis (LDA) effect size (LEfSe) method was used to investigate bacterial community at the phylum level. LDA score higher than 2 indicates a higher relative abundance in the corresponding group than in other groups. ASV, amplicon sequence variant; OTU, operational taxonomic unit; PCoA, principal coordinates analysis. The meaning of the asterisk symbol indicates significant difference. (P < 0.05).

The relative abundance of microbiota was severely disturbed in the MOD group. It was observed that the relative abundance of phyla *Firmicutes* was significantly decreased while the phyla *Bacteroidetes* and *Proteobacteria* were markedly increased (**Figure 7E**), which was similar to the findings by Guo et al. (24). *L. paracasei* X11 administration attenuated HUA-induced reduction in *Firmicutes* and addiction in *Bacteroidetes* (**Figures 7F, G**). The ratio of *Bacteroidetes* to *Firmicutes* (Bac/Firm Ratio), in which disproportion could lead to metabolic syndrome such as obesity and diabetes (27), was recovered nearly to the level in CON mice by *L. paracasei* X11 therapy (**Figure 7H**). At the genus level, the results showed that the relative abundance of *Muribaculaceae* and *Bacteroides* was increased after HUA modeling, while that of *Lachnospiraceae*_NK4A136_group and *Alistipes* decreased (**Figure 7I**). In addition, the relative abundance of *Lactobacillus* in the X11 group was higher than that of the other three groups (**Figure 7J**), which indicated that *L. paracasei* X11 had a positive effect on gut microbiota. It was worth noting that the promising probiotic *Faecalibaculum* was significantly enriched in the X11 mice (**Figures 7K, L**), which played an antitumor role by producing short-chain fatty acids (SCFAs) (28). These results suggested that *L. paracasei* X11 could shape the intestinal microbiota of the HUA mice and alleviate symptoms.

## Discussion

HUA is a purine metabolic disorder disease that persists in arising health problems all over the world (2). With changes in lifestyle and dietary patterns, the prevalence of HUA is influenced by a variety of innate or acquired factors, such as genes, high purine food intake, stress anxiety, and sub-healthy physical condition (5). Due to the drawbacks of existing treatment for HUA (17), UA-inhibiting or UA-excreting drugs may increase the associated risk of inducing kidney stones and cause all-cause cardiac death. Therefore, it is gaining much attention to regulate the UA metabolism through mild probiotic intestinal therapy. It was reported that probiotic supplements could prevent the accumulation of UA successfully. Wu et al. found that *Limosilactobacillus fermentum* JL-3 reduced UA levels in mice and regulated the structure of gut microbial (19). Kuo et al. reported that *Lactobacillus reuteri* TSR332 and *Lactobacillus fermentum* TSF331 stabilized serum UA levels and prevented HUA in rats (29). In addition, prophylactic treatment with *Lactobacillus brevis* DM9218-A decreased UA concentration in HUA rats (30). Thus, probiotics with UA-lowering ability might be a promising strategy for the treatment of HUA.

Nucleotides, nucleosides, purine, and trioxypurine were involved in the metabolic pathway of UA. In the report of Wu et al, *Li. fermentum* JL-3 was screened out by using UA as a target and could degrade UA by 40.90% in 24 h (19). In our study, these four metabolites were selected as targets to screen probiotics with UA-lowering ability. Among 20 candidate strains, *L. paracasei* X11 exhibited excellent assimilation capability and could assimilate nucleotides (100%), nucleosides (100%), purine (83.25%), and trioxypurine (80.42%) within 30 min (*p* < 0.05). Urate oxidase could degrade relatively insoluble UA to highly soluble allantoin, which exists in non-primate mammals and lower primates while lost in humans and higher primates in evolution. Therefore, it is difficult to establish a stable HUA animal model due to the expression of urate oxidase in mice. Presently, peritoneal injection of potassium oxazinate with long-term high-purine diets was chosen to induce HUA (31). However, injection of potassium oxazinate every day caused side effects of diarrhea, hematochezia, and even death of mice. In our study, it was found that intermittent injection of potassium oxazinate in the first week not only could avoid the above side effects but also could establish the hyperuricemia model successfully. After 14 days of modeling, the serum levels of UA, BUN, XOD, and Cr in the MOD group were 1.5–2-fold higher than those of the CON group. At the same time, the mice in the MOD group showed symptoms of listlessness and weight loss, which was in accordance with the reports of Wu et al. (19). Studies have shown that ALLO was selected as a positive control because it could reduce serum UA by inhibiting UA synthesis in the liver (8). Under 14 days of intragastric administration, compared with those of the MOD group, the body weight and the serum lipid index of the X11 group were recovered to a normal level significantly. Though serum UA, BUN, and XOD were downregulated in the ADC group, the weight loss was more serious, and the Cr reflecting renal function was further increased and higher than that of the MOD group. A similar pattern was observed in histopathological H&E micrographs, which demonstrated that *L. paracasei* X11 could reduce the injury to the liver, kidney, and intestine in HUA mice. In addition, it aggravated the damage to the kidney and intestinal tract after ALLO treatment. LPS, IL-1β, and TNF-α are important inflammation biomarkers, and MDA is commonly used as an indicator of peroxidation. Changes in LPS, IL-1β, TNF-α, and MDA can reflect the state of the body’s inflammatory reaction (25). In our study, the results showed that *L. paracasei* X11 could alleviate abnormalities in proinflammatory factors and improve the antioxidant activity. The inflammation symptoms were relieved, and the occurrence and development of HUA were attenuated, which was consistent with the effects of *Li. fermentum* JL-3 (19) and *L. brevis* DM9218 (32).

ADA and XOD are key enzymes involved in the production of hepatic UA. It was reported that lactic acid bacteria could relieve HUA by suppressing XOD activity *via* an SCFA-dependent mechanism (33). In our study, we found that *L. paracasei* X11 could downregulate the activity of ADA and XOD in the liver significantly. The kidney is the main organ of UA excretion, and about 2/3 of UA was excreted by the kidney. Renal UA reabsorption transporters GLUT9, NPT1, and excretory transporter URAT1 played important roles in mediating UA excretion (4, 16). In our experiment, it was observed that the expressions of GLUT9 and NPT1 were increased in the MOD group, but oral administration of *L. paracasei* X11 decreased these excessive expressions to a normal level. It suggested that renal UA reabsorption aggravated in HUA while *L. paracasei* X11 ameliorated this phenomenon and promoted excretion. Similar studies have confirmed that altering transporter expression could regulate human urate excretion and thereby ameliorate HUA (34).

The gut microbiota is another crucial factor in the etiopathogenesis of HUA. It was reported that HUA caused an imbalance of gut microbiota, including an increase in pathogenic bacteria and a decrease in gut microbial diversity (24). In our previous study, it was observed that probiotics could alter gut microbiome composition in the absence of gut inflammation (25). In this study, the effect of *L. paracasei* X11 on gut microbiota in HUA was explored. Surprisingly, it was found that *L. paracasei* X11 reshaped and restored the composition of gut microbiota in HUA mice. The diversity and the abundance of gut microbiota in the MOD group were largely lessened compared to those of the CON group, which were moderated and improved by *L. paracasei* X11 administration. Furthermore, the α-diversity and β-diversity of microbiota could be used to predict the activation of cells and dynamic balance of gut flora (35), which became a normal microbial community in the X11 group. At the phylum level, *L. paracasei* X11 alleviated the relative abundance of *Bacteroidetes* and *Proteobacteria* and adjusted the proportion of *Bacteroidetes* to *Firmicutes* to the normal level. At the genus level, the relative abundance of *Lactobacillus* was significantly increased in the CON group compared with the other 3 groups. Particularly, *L. paracasei* X11 treatment increased the abundance of some beneficial gut microbes, such as *Faecalibaculum*, which was reported to produce SCFAs to ameliorate tumor progression (28). More importantly, it was reported that there was a strong correlation between the gut microbiota and inflammatory cytokines of the immune-inflammatory pathways (35), which was consistent with the phenomena observed in our study. These results could be inferred that *L. paracasei* X11 might regulate intestinal immune homeostasis *via* the gut microbiota in HUA mice. The exact mechanisms needed to be further investigated.

In conclusion, it was found that *L. paracasei* X11 from Chinese traditional fermented food exhibited high UA-lowering ability *in vitro* and could downregulate serum biochemical indices, restore organ damage, and alleviate the inflammatory response of HUA mouse models. It was confirmed that *L. paracasei* X11 could regulate metabolism enzyme and transporter expression to normal levels. Furthermore, *L. paracasei* X11 had a potential effect to recover the structure and function of the gut microbial community. These findings suggested that *L. paracasei* X11 had the potential to be developed as a novel probiotic to ameliorate HUA.

## Data Availability Statement

The datasets presented in this study can be found in online repositories. The name of the repository and accession number can be found below: NCBI Sequence Read Archive; PRJNA838715.

## Ethics Statement

All experimental processes were approved by the Animal Ethics Committee of Ocean University of China (Permission number: SPXY2022011201).

## Author Contributions

Conceptualization: HY. Methodology: JC, QL, and HH. Formal analysis: JC, QL, and TW. Software: JC and HH. Supervision: HY. Data curation: JC and QL. Writing—original draft preparation: JC, QL, and HH. Writing—review and editing: HY. Visualization: YB and XT. Project administration: HY. Funding acquisition: HY. All authors contributed to the article and approved the submitted version.

## Funding

This work was supported by the National Natural Science Foundation of China (Nos. 32172180, 31771988).

## Conflict of Interest

The authors declare that the research was conducted in the absence of any commercial or financial relationships that could be construed as a potential conflict of interest.

## Publisher’s Note

All claims expressed in this article are solely those of the authors and do not necessarily represent those of their affiliated organizations, or those of the publisher, the editors and the reviewers. Any product that may be evaluated in this article, or claim that may be made by its manufacturer, is not guaranteed or endorsed by the publisher.
